# A Study on Early Death Prognosis Model in Adult Patients with Secondary Hemophagocytic Lymphohistiocytosis

**DOI:** 10.1155/2022/6704859

**Published:** 2022-07-01

**Authors:** Ruoxi Zhang, Tingting Cui, Lingbo He, Menghan Liu, Zhengjie Hua, Zhao Wang, Yini Wang

**Affiliations:** ^1^Department of Hematology, Beijing Friendship Hospital, Capital Medical University, Beijing, China; ^2^Department of General Medicine, Beijing Friendship Hospital, Capital Medical University, Beijing, China

## Abstract

**Background:**

The mortality risks for secondary hemophagocytic lymphohistiocytosis in the induction stage and investigated prognostic factors need to be further discussed.

**Objective:**

The aim of this study is to establish a clinical model for predicting early death in adult patients with secondary hemophagocytic lymphohistiocytosis. *Design, Participants, and Main Measures*. The baseline characteristics, laboratory examination results, and 8-week survival rate of 139 adult sHLH patients diagnosed from January 2018 to December 2018 were analyzed retrospectively, and a prognostic model was constructed with low-risk (score 0–2), medium-risk (score 3), and high-risk (score ≥ 4) as parameters. *Key Results*. Univariate analysis confirmed that early death was not related to the type of HLH but significantly related to the patient's response to first-line treatment. The peripheral blood cell count was significantly decreased, C-reactive protein was higher, glutamyl transpeptidase and total bilirubin were higher, albumin was significantly lower, urea nitrogen was higher, hypocalcemia and hyponatremia, deep organ hemorrhage and D-dimer increased, cardiac function damage and HLH central involvement, sCD25 increased, and EB virus infection were predictive factors of early death. In the multivariate model, patients' response to first-line treatment was a good predictor of overall survival, and hypocalcemia and deep organ bleeding were associated with poor survival. The risk factors were scored and graded according to the risk ratio. The 8-week overall survival rates of the low-risk group (82 cases), medium-risk group (36 cases), and high-risk group (21 cases) were 85.4%, 52.8%, and 23.8%, respectively (*P* < 0.001).

**Conclusions:**

The early death of sHLH patients is closely related to some laboratory examination results. Attention should be paid to identify high-risk patients, choose effective first-line induction therapy, achieve deep remission as soon as possible, prevent deep organ bleeding, correct electrolyte disorders, and improve the early survival rate of sHLH patients.

## 1. Introduction

Hemophagocytic lymphohistiocytosis (HLH) is a kind of excessive inflammatory reaction caused by hereditary or acquired immune dysfunction, which leads to excessive activation of T cells and macrophages and produces a large number of inflammatory factors to infiltrate multiple organs and tissues, which is life-threatening. HLH used to be considered a pediatric disease, but with the worldwide reports and gradual recognition of the onset of HLH in adulthood, it has been confirmed that it can occur at any age.

Active HLH has rapid progress and high mortality. In the 1980s, the median survival time of HLH was only 1–2 months, and the [1] 1-year overall survival rate was only 5%. Until the birth of the world's first clinical study on HLH treatment, HLH-94 significantly increased the induced remission rate of HLH from less than 10% in the past to about 70%, and the subsequent allogeneic hematopoietic stem cell transplantation (allo-HSCT) benefited nearly 50% of patients [2]. At present, allo-HSCT has been recognized as the only cure for HLH [3], which can overcome the impact of different underlying diseases and clinical conditions of HLH on survival and prognosis [4]. However, the results of both HLH-94 and HLH-04 clinical studies show that although allo-HSCT changes the long-term survival of HLH, the peak of death is concentrated in the first 8 weeks of induction therapy [2, 5].

According to the etiology, HLH can be divided into primary HLH and secondary HLH. SHLH is induced by a variety of pathological factors, mainly malignant tumor, infection, and autoimmune disease. The disease of sHLH is progressing rapidly and the mortality is high. Researchers have been trying to explore the prognostic markers of HLH. A series of studies have reported the prognostic factors affecting the long-term survival of patients with HLH [6–8]. However, the related prognostic factors and risk stratification of early death in adult sHLH need to be further discussed.

## 2. Methods

### 2.1. Clinical Data

This study retrospectively analyzed the clinical data of adult patients (age ≥18 years) who received systematic treatment in Beijing Friendship Hospital affiliated to Capital Medical University from January 2018 to December 2018. All patients met the diagnostic criteria of HLH-2004 that are [9]: (1) known genetic defects were confirmed by molecular biological examination; (2) 5 of the following 8 indexes were consistent: 1 fever, lasting >7 days and body temperature ≥38.5°C. (2) Splenomegaly; (3) hemocytopenia (involving two or three lines of peripheral blood): hemoglobin <90 g/*L*, platelet <100 × 10^9^/*L*, and neutrophils <1.0 × 10^9^/*L*, which is not caused by decreased hematopoietic function of the bone marrow; (4) hypertriglyceridemia and/or hypofibrinogenemia: triglyceride >3 mmol/L or 3 standard deviations higher than 3 standard deviations of the same age, fibrinogen <1.5 g/L or lower than 3 standard deviations of the same age. (5) Hemophagy was found in bone marrow, liver, spleen, or lymph nodes. (6) The activity of natural killer (NK) cells was decreased or absent. (7) Ferritin ≥500 *μ* g/*L*, (8) soluble interleukin-2 receptor (sCD25) increased, and secondary HLH was identified by systemic venereal disease.

### 2.2. Research and Design

The clinical parameters of the patients were collected, including the clinical indexes related to the diagnosis of HLH, liver function, renal function, cardiac function, blood coagulation function, electrolyte, central involvement, induction treatment effect, and so on. The survival rate within 8 weeks after treatment was analyzed, and a prognostic model was constructed with low risk, medium risk, and high risk as parameters. Early death is defined as death within 8 weeks after diagnosis.

### 2.3. Statistical Analysis

Statistical analysis was conducted using SPSS (version 21.0, Chicago, Illinois, USA) and GraphPad Prism 6 (La Jolla, California). Through standard descriptive statistics, the characteristics of patients were summarized as the median ± quartile. The area (AUC) value under the curve and the confidence interval (CI) were used to calculate the best survival cutoff value by using ROC analysis of subjects' working characteristics. Estimation of OS by the Kaplan–Meier method and the difference between survival curves was estimated by Logrank test in univariate analysis. Multivariate Cox analysis (risk ratio (HR) and 95% confidence interval) was used to identify independent prognostic variables of OS and calculate survival risk. *P* < 0.05 is considered to be statistically significant.

## 3. Results

### 3.1. Basic Clinical Features

This study retrospectively analyzed 139 newly diagnosed adult cases of sHLH, of which 80 were males and 59 were females, with a median age of 38 years (28–51 years). Among them, 63 cases of EBV-related HLH, 33 cases of tumor-related HLH, and 43 cases of autoimmune diseases were identified. Efficacy was assessed within 2 to 4 weeks after initial induction therapy (HLH-1994) in all enrolled patients, and the main indicators of efficacy evaluation included sCD25, ferritin, blood count, triacylglycerol, hemophagocytosis, and level of consciousness (in those with CNS-HLH). Complete Response (CR): all of the above indicators returned to the normal range. Partial response(PR): ≥2 symptoms/laboratory indicators improved by more than 25%, and individual indicators needed to meet the following criteria: (1) sCD25 levels decreased by more than 1/3; (2) ferritin and triacylglycerol decreased by more than 25%; (3) without blood transfusion: neutrophil <0.5 × 10^9^/L, need to rise 100% and >500 × 10^9^/L; neutrophils 0.5–2 × 10^9^/L, need to increase by 100% and return to normal; (4) ALT >400 U/L, need to decrease by more than 50%. The overall response rate was 69.1%, of which 46 patients (33.1%) reached CR, 50 patients (36.0%) achieved partial response PR, and 43 patients (30.9%) did not respond to the initial treatment (NR) and then changed the treatment regimen (DEP). 45 patients died within 8 weeks of diagnosis, accounting for 32.4% of the total cases.

### 3.2. Characteristics of Clinical Parameters in Diagnosis of HLH

Analyzing the clinical parameters related to the diagnosis of HLH, fever was present in almost all patients, with a body temperature >38.5°C accounted for 95.7%, and 84.8% of patients with high fever above 39°C. Spleen enlargement occurs in 79.7% of patients, while liver enlargement occurs in only 29% of patients. In peripheral hemocytopenia, leukopenia, and thrombocytopenia are more common, accounting for about 65.5% and 72.7%, respectively. Patients with triglycerides >3 mmol/L and fibrinogen <1.5 g/L accounted for 37.2% and 44.9%, respectively. Hemophagocytosis was found in the bone marrow in 81% of patients, and elevated ferritin and sCD25 were the most prominent clinical indicators of HLH, with abnormality rates of 94.9% and 96%, respectively. HLH central involvement presents in 22.1% of patients. HLH central nervous system involvement (CNS-HLH) is characterized by neurological and/or psychiatric symptoms (e.g., irritability, convulsions, epilepsy, meningeal irritation, altered consciousness, ataxia, hemiplegia, etc.), CNS imaging abnormalities (MR/suggesting changes in the brain parenchyma or meninges), and cerebrospinal fluid (CSF) abnormalities [CSF cell >5 *μ*L, and/or elevated protein >35 g/L). When one or more of these signs are present in patients with HLH, CNS-HLH should be considered.

By analyzing other parameters that reflect the basic state of the patient, it can be found that about 70% of the patients have abnormal liver function (defined in this paper as transaminase or bilirubin more than 2 times the normal upper limit). The abnormal rates of glutamic pyruvic transaminase, glutamic oxaloacetic transaminase, and bilirubin were 54.3%, 59.7%, and 36%, respectively. The abnormal rate of lactate dehydrogenase is as high as 86%; about half of the patients have significant hypoalbuminemia. Hypocalcemia and hyponatremia were the most common in patients with electrolyte disorders, with 58.3% and 42.4% of patients complicated with hypokalemia, respectively. Abnormal blood coagulation was seen in 75.5% of patients, of which 20.1% were complicated by bleeding of deep organs (including digestive tract, lung, and center). Cardiac dysfunction was seen in 20.9% of patients.

The clinical parameters of patients with HLH are shown in Table 1.

### 3.3. HLH Early Death Prediction Model

Univariate analysis showed that decreased peripheral blood cell count, high C-reactive protein, high glutamyl transpeptidase and total bilirubin, significantly decreased albumin, high urea nitrogen, hypocalcemia and hyponatremia, deep organ hemorrhage and elevated D-dimer, cardiac function damage and HLH central involvement, EBV infection, and elevated SCD25 were associated with poor prognosis. The response of patients to first-line treatment had a significant impact on the survival rate during the induction treatment period, while the primary disease leading to HLH had no significant effect on the early survival of patients (Prun0.144). In the multivariate COX model, deep visceral hemorrhage (HR = 2.746, 95% CI 1.041–7.242), first-line induction therapy (HR = 0.122 and 0.291 pc 95% CI 0.029–0.509 and 0.088–0.960) and hypocalcemia (HR = 0.305, 95% CI 0.094–0.986) were independent prognostic factors (Table 2). The risk factors were scored according to the risk ratio: deep organ hemorrhage (score 2), the effect of first-line induction therapy (PR = score 2, NR = score 3), and hypocalcemia <1.8 mmol/L (score 1). Use these variables for risk scoring and stratification. The 8-week overall survival rates of 82 patients in the low-risk group (score 0–2), 36 patients in the medium-risk group (score 3) and 21 patients in the high-risk group (score ≥4) were 85.4%, 52.8%, and 23.8%, respectively (Figure 1).

## 4. Discussion

HLH is a rapidly progressive and highly fatal disease that occurs in all age groups. According to the underlying etiology, HLH can be divided into two categories: primary and secondary. Primary HLH has genetic defects, while secondary HLH is caused by many underlying diseases, the most common causes of which include infection, malignant tumors and autoimmune diseases [10]. The treatment strategy of HLH is divided into two main aspects: the short-term strategy is mainly to control the excessive inflammatory state, and the long-term strategy is to correct the potential immune deficiency and control the primary disease, which means that the potential etiology of HLH strongly affects the prognosis of HLH, and the prognosis of tumor-related HLH is the worst [11].

The results of two famous clinical studies on HLH, HLH-94 and HLH-2004, as well as other clinical observation studies on different types of HLH, believe that allo-HSCT is the only means to overcome the impact of primary diseases on the long-term survival of HLH patients and improve the overall survival rate [12–14]. However, a large sample of clinical studies also found that in the group of patients who did not receive allo-HSCT, the death rate of 2/3 was mainly concentrated in the first 8 weeks of the induction treatment period after diagnosis, especially in patients who died in 6–8 weeks because of refractory disease progression and organ failure, while the peak of death of 1/3 was concentrated in those who had not received allo-HSCT 120 days after diagnosis [5]. Identifying high-risk factors for death in the first 8 weeks of the induction treatment period, identifying patients at high risk of early death, and providing timely stratified individualized treatment are key factors in reducing mortality in patients with HLH. However, the available studies have only explored the prognostic factors affecting the long-term survival of HLH patients and have not explored the prognostic factors and risk stratification associated with early mortality in adults with sHLH. Therefore, there is a need to investigate the high-risk factors that lead to death in HLH patients during the induction phase to help the clinic identify high-risk patients early and provide a basis for developing stratified individualized treatment.

In this study, the clinical parameters of adult sHLH were analyzed and compared in detail. From the univariate analysis, the early death of sHLH patients was not closely related to the type of HLH, which also indicated that HLH had something in common under a wide range of clinical conditions—excessive pathological inflammatory reaction [15]. The first step to improve the survival rate was to control the inflammatory state of over-activation of the body. Instead of dwelling on the primary disease hidden behind HLH, we should not delay clinical treatment in order to wait for the test results [16]. Among the indexes related to the diagnosis of HLH, the decrease of peripheral blood cell count, the decrease of fibrinogen, and the central involvement of sCD25 and HLH were closely related to early death. Other diagnostic indexes had no significant effect on survival within 8 weeks. Among the other indicators that reflect the basic state of the body at the time of diagnosis, a number of clinical parameters are related to early death, such as high levels of glutamyl transpeptidase and total bilirubin reflecting liver function, azotemia reflecting renal function, and increased C-reactive protein, which reflects that the body may be complicated with infection. Nutritional status and water-electrolyte balance indicators are related to multiple organ dysfunctions, such as abnormal blood coagulation, cardiac function damage, hypoalbuminemia, hypocalcemia, and hyponatremia. These results also reflect the pathophysiological mechanism of HLH-excessive activation of T cells and macrophages, the production of a large number of inflammatory factors infiltrating multiple organs. We speculate that the risk of early death in patients with HLH comes more from the damage to organ function and the effect of HLH on the internal environment of the body. When the patient has more complications, it means that the treatment is more difficult and the window period is shorter.

After further multivariate regression analysis, we can see that the independent risk factors that really affect the early survival rate of adult sHLH are patients' blood calcium, the presence of deep organ bleeding and patients' response to first-line induction therapy. The selection of effective first-line induction therapy can to a large extent improve the serious and bad basic condition of patients in the early stage of treatment and create conditions for survival and further clear diagnosis of potential diseases and targeted treatment. Bleeding in deep organs is the main risk of acute death before treatment takes effect [17, 18]. As a coagulation factor, serum calcium is a risk factor for bleeding events in patients.

A series of studies have reported on prognostic factors for HLH, most of which have been on prognostic factors for long-term survival. A study on adult nonmalignant tumor-related sHLH prognostic factors found that response to EB virus infection, advanced age, thrombocytopenia, and methemoglobinemia were associated with poor prognosis at 8 weeks of treatment [6]. In another study aimed at developing a model to assess the six-month prognosis of adult HLH patients, three laboratory markers were identified as independent risk factors: ferritin, platelets, and alanine aminotransferase [19]. And a study suggested that gender, platelet count, albumin, alanine aminotransferase, and treatment regimens were independent prognostic factors for HLH in adults [20]. The subjects of our study are adult secondary HLH patients, which reflects the early clinical characteristics of the adult sHLH population. In univariate analysis, the results are basically consistent with the above results, but there are differences after multivariate regression, which may be due to the fact that this study analyzes the prognostic factors that affect the long-term survival of HLH patients, while this study focuses on the influencing factors of early death. The long-term survival of patients with HLH is related to the control of the primary disease, while early survival is related to excessive inflammation. The above studies did not include NK cell activity, sCD25, or CRP, and did not analyze patients' overactive inflammatory states. Another study analyzing 5-year survival risk factors in patients with adult sHLH reported that males, APTT >36 s, LDH>1000 U/L, and CRP >100 mg/L were risk factors for prognosis in patients with HLH [21]. The study analyzed the prognostic factors that affect the long-term survival of patients with HLH as the same, which did not include electrolytes such as Ca^2+^ and Na^+^. In our study, hypocalcemia and hyponatremia were closely related to early death, and we speculate that the risk of early death in patients with HLH may be related to the effects of HLH on the body's internal environment. However, in the study on the prognostic factors for early death from HLH in adults, malignancy, hypertriglyceridemia, thrombocytopenia, elevated lactate dehydrogenase, prolonged APTT, and advanced age were risk factors [22].The results of our study are quite different from those of this adult cohort study. The main reason is that the adult HLH study ignores the direct and important impact of effective first-line induction therapy on survival outcomes. In fact, the international mainstream academic point of view also believes that the survival rate of the induction period is closely related to the effective rate of treatment. If patients have no obvious response to treatment within 2–3 weeks, they should consider changing the treatment regimen [23]. In our study, not only did the response rate of HLH patients in first-line induction therapy reach 69.1% but also some nonresponsive patients got disease remission and prolonged survival time after changing salvage treatment in time. On this basis, the adverse prognostic factors screened out may more objectively reflect the clinical risk stratification of HLH.

In addition, this study also established a prognostic model for the early death of adult sHLH. According to the risk ratio, three independent risk factors affecting the early survival rate of adult sHLH were scored and stratified, and the patients were divided into three groups: low risk, medium risk, and high risk. There was a significant difference in the overall survival rate of 8 weeks. Through the risk stratification of the clinical parameters at the time of diagnosis and the survival rate within 8 weeks after treatment, it is helpful to identify high-risk patients early and carry out targeted treatment in time.

In this study, we analyzed the clinical parameters of 139 adult sHLH patients who died during the induction treatment period and evaluated prognostic factors for treatment response and survival outcomes, and found that patient response to first-line therapy was a good predictor of overall survival, and hypocalcemia and deep organ bleeding were associated with poorer survival, and finally, we developed a prognostic model using risk stratification based on the predictors that provides a basis to help clinical identification of high-risk factors for early death and timely targeted treatment.

Our study has certain limitations. This is a retrospective research and inevitably there are missing values, so we analyzed the missing pattern of missing values and performed multiple interpolations, which may cause some bias to the results. Since only a single-center retrospective study was conducted, our prognostic model has not been validated by a larger study, and therefore, further multicenter and prospective studies are needed to confirm the clinical value of the model to improve early survival in patients with sHLH. It has been suggested that the InfusedHeart Framework can be extended to solve various cardiac-risk classification issues [24]. The InfusedHeart Framework provides a new approach to the evaluation of cardiac impairment as an indicator, and we will try to apply it to the evaluation of cardiac impairment in our follow-up study.

## 5. Conclusion and Future Work

Early death in adults with sHLH is closely related to the basal state of the organism and the impaired organ function of the patient before treatment. In future clinical work, the prognostic model should be applied to stratify patients diagnosed with sHLH at risk, identify patients at high risk of death early, target early death predictors, carry out timely treatment, select effective first-line induction therapy, achieve deep remission as early as possible, prevent deep organ bleeding, maintain body electrolyte balance, and improve the early survival rate of patients with sHLH.

## Figures and Tables

**Figure 1:** The 8-week overall survival rates of 82 patients in the low-risk group(score 0–2), 36 patients in the medium-risk group(score 3) and 21 patients in the high-risk group (score≥ 4) were 85.4%, 52.8% and 23.8%.

**Table 1:** Clinical characteristics of 139 patients with sHLH.

Characteristics	Median	Quartile
WBC (×10^9^/L)	2.22	1.2–4.59
HGB (g/L)	89	78–109
PLT (×10^9^/L)	54	27–114
CRP (mg/L)	22	5–78.05
ALT (U/L)	94	42–198.25
AST (U/L)	90.9	40.8–220.8
LDH (U/L)	529.5	314.85–1069.5
*γ*-GT (U/L)	116	50–270
ALP (U/L)	156	93–337
TBil (umol/L)	22.1	15.12–54
Alb (g/L)	30	24.1–34
Glb (g/L)	25.9	20.8–30.7
Scr (umol/L)	60.3	50.9–76.3
BUN (mmol/L)	5.23	4.03–7.29
TG (mmol/L)	2.48	1.77–3.55
K (mmol/L)	3.91	3.67–4.25
Ca (mmol/L)	2.04	1.91–2.15
Na (mmol/L)	135.9	132.1–138.8
CO2CP	24.4	22.7–26.7
Fg (g/L)	1.675	1.1475–3.28
SF (ng/ml)	2385	1286.75–11409.95
sCD25 (pg/ml)	26271	15957.65–40939.75
NK cell activity (%)	14.675	12.97–16.29
CD107a (%)	13.15	8.47–20.31
EBV-DNA (copy/ml)	9.9 *E* + 002	0–4.7475 *E* + 004
D-dimer (mg/L)	2.6	1.1–8.2

WBC, white blood cell; HBG, hemoglobin; PLT, platelet; CRP, C-reactive protein; ALT, alanine transferase; AST, aspartate aminotransferase; LDH, lactic dehydrogenase;,*γ*-GT: *γ*-glutamyl transpeptidase; ALP, alkaline phosphatase; Fg, fibrinogen; CO2CP, carbon dioxide combining power; NK cell activity, natural killer cell activity; EBV, Epstein-Barr virus.

**Table 2:** Prognostic factors of overall survival of 139 patients with sHLH.

Univariate analysis			Multivariate analysis		
	8-week OS	*P*	HR	*P*	95% CI
WBC (×10^9^/L)		0.024^*∗∗*^			
<2	57.6%				
HGB (g/L)		<0.001^*∗∗*^			
<80	46.3%				
PLT (×10^9^/L)		0.003^*∗∗*^			
<30	50.0%				
CRP (mg/L)		0.023^*∗∗*^			
>25	77.1%				
*γ*-GT (U/L)		0.05			
>200	73.9%				
TBil (umol/L)		0.015^*∗∗*^			
>20	79.3%				
Alb (g/L)		0.005^*∗∗*^			
<30	58.0%				
BUN (mmol/L)		0.015^*∗∗*^			
>6	74.7%				
Ca (mmol/L)		<0.001^*∗∗*^	0.305	0.047^*∗*^	0.094-0.986
<1.8	30.0%				
Na (mmol/L)		0.033^*∗∗*^			
<135	57.4%				
sCD25 (pg/ml)		0.005^*∗∗*^			
>30000	82.1%				
EBV (copy/ml）		0.008^*∗∗*^			
> 6.5E+003	76.7%				
D-Dimer (mg/L)		0.002^*∗∗*^			
>3.6	77.5%				
Cardiac Impairment		0.003^*∗∗*^			
Yes	48.3%				
Visceral Hemorrhage		0.003^*∗∗*^	2.746	0.041^*∗*^	1.041–7.242
Yes	46.4%				
CNS Involvement		0.001^*∗∗*^			
Yes	44.8%				
response to induction therapy		<0.001^*∗∗*^	0.122	0.004^*∗∗*^	0.029–0.509
CR	89.1%		0.291	0.043^*∗*^	0.088–0.960
PR	68%				
NR	44.2%				

Abbreviation: OS, overall survival; HR, hazard ratio; ^*∗*^ *<* 0.05; ^*∗∗*^*P* *<* 0.01, variables used in multivariate analysis were selected after excluding significant correlations: Ca, visceral hemorrhage, response to induction therapy.

## Data Availability

The datasets used during the current study are available from the corresponding author on request.
